# Effectiveness of a therapeutic patient education program in improving cancer pain management: EFFADOL, a stepped-wedge randomised controlled trial

**DOI:** 10.1186/s12885-019-5836-5

**Published:** 2019-07-08

**Authors:** Virginie Prevost, Natacha Heutte, Alexandra Leconte, Idlir Licaj, Claire Delorme, Bénédicte Clarisse, and on behalf of the EFFADOL-Group

**Affiliations:** 1 University of Normandy, 14000 Caen, France; 2 UMR 1086 INSERM « ANTICIPE », Centre François Baclesse, 14000 Caen, France; 3 Clinical Research Department, Centre François Baclesse, 14000 Caen, France; 4 Bayeux Hospital, 14400 Bayeux, France; 5 Regional Pain Network for Lower Normandy, 14400 Bayeux, France

**Keywords:** Pain management, Pain cancer, Patient education, Stepped-wedge randomised controlled trial, Quality of life

## Abstract

**Background:**

Despite numerous guidelines, nearly one of two patients with cancer pain remains undertreated, thereby affecting their quality of life. Active patient involvement through Therapeutic Patient Education (TPE) is considered as a relevant strategy to overcoming hurdles in pain management. The aim of the EFFADOL study is to assess the effectiveness of a TPE program in improving cancer pain management.

**Methods/design:**

The EFFADOL study is a stepped-wedge randomised controlled trial. A total of 260 cancer patients with unbalanced background pain will be randomised over the institutional level, i.e. stepped-wedge cluster design. Six clusters will be formed, one at the regional level of “Basse-Normandie” for patients receiving the educational approach by health providers already trained to TPE. Then, five additional centers will be gradually included at the national level, making it possible to compare the “conventional” management of pain (before medical staff training to TPE) with the educational approach (after being trained). The main study parameter is pain interference on daily life assessed with the self-administrated and validated Brief Pain Inventory questionnaire. Secondary objectives comprised the evaluation of patients’ adherence to pain education program, the description of pain intensity, pain relief, analgesic adherence and pain emotional impact. Educational dimension of the program will be evaluated through the patients’ acquisition of knowledge and skills about their pain and treatment as well as their self-efficacy to participate actively in pain management. The patient’s feeling of pain changes will be measured. Finally, the satisfaction of participants and educators will be reported. We hypothetise active involvement of patients in TPE will lead to an improved pain management compared to standard care.

**Discussion:**

Analyzing the impact of a TPE program in cancer pain patients will improve their pain management and quality of life. We expect that the dissemination of our project educational approach through the French territory will be accompanied by long term change in clinical practices with mutual benefit to patients and caregiver-educators.

**Trial registration:**

NCT03297723, registered: 09/28/2017.

Protocol version: Version n°1.1 dated from 2016/09/08.

## Background

Pain remains a prevalent symptom in patients with cancer despite the availability of opioids and current guidelines [1]. Based on a recently updated meta-analysis, pain prevalence is indeed 55% during anticancer treatment [2]. Pain, when it is not effectively treated and relieved, has a severe impact on quality of life [3]. Greco et al. [4] reported that 31.8% of cancer patients still do not receive analgesic treatment proportional to their pain intensity.

The management of cancer pain encounters various obstacles, including patient-related barriers [5, 6] such as the lack of knowledge and representations of patients about pain and its treatment. Barriers include widespread misconceptions about opioid use, underestimation of pain, and non-adherence to treatment [7].

Active patient involvement through Therapeutic Patient Education (TPE) is considered as a relevant strategy to overcoming obstacles in cancer pain management [7]. TPE, as defined by the World Health Organization (WHO, [8]), aims at enabling patients to develop skills to achieve optimal cancer pain control and therefore improve their QoL. TPE programs for pain management have been developed in recent years and the number of published studies evaluating Pain Education Programs (PEP) and establishing the most efficient programs to date has substantially increased, as highlighted in our recent literature review [9]. In particular, Oldenmenger’s systematic review [10] recently performed on 26 Randomised Controlled Trials (RCT) totalling 4735 patients, shows that PEP may result in improvements of relevant patient-reported outcomes. Adam et al. [11] analysed 34 RCT and 8 systematic reviews (including 3 meta-analyses [12–14]) in the field of cancer pain covering nearly 40 years. Reviews showed a slight but statistically significant effect of PEP on knowledge about pain and attitudes towards it, as well as a decrease in pain intensity as reported by patients. Even if there are some evidences of the benefit of PEP on improving pain management, educational interventions are complex. This still raised many issues, including the optimal choice for types of intervention, study designs, and outcome measurements.

In this context and according to the regional health policy, we have undertaken an extensive five-step research program, called EFFADOL (“*Ensemble, Faire FAce à la DOuLeur”*), structured in 5 successive phases, each of them briefly described in the paper developing the EFFADOL combined approach from practice to research [15]. Health professionals were first trained in TPE (step 1). We identified patients’ and relatives’ needs with regard to pain (step 2, [16] prior to design a PEP dedicated on cancer pain (step 3). The PEP evaluation includes an assessment of its feasibility, quality and transferability at the regional level (step 4) and of its effectiveness at the French level through an interventional comparative randomisation (step 5).

Thus, the research steps (2, 4, and 5) complement the implementation of the PEP (Step 3) answering to the ethical and regulatory requirements of TPE that place emphasis on the importance given upstream to the identification of patient expectations and needs (Step 2,) and downstream on that of evaluation (Steps 4 and 5). The proposed strategy, beyond these requirements, confers a prospective experimental dimension to the whole project in order to answer the following research question: does TPE allow patients suffering from cancer to manage their pain better on a daily basis? We herein detail the methodology of the evaluation step 5 aiming to evaluate the effectiveness of our PEP in improving pain management among cancer patients.

### Objectives

The main objective of this study (Step 5 of the EFFADOL program) is to assess the PEP effectiveness on patients’ pain through pain interference with daily life as main judgement criterion.

We will further evaluate the proportion of patients adhering to the whole PEP at the Basse-Normandie scale (Step 4), and then at the national level after medical staff being trained to TPE.

Other secondary objectives, dealing with the overall effect of pain education on pain management, aim:

- To assess pain intensity, pain relief, and emotional impact.

- To assess patients’ skills and knowledge.

- To evaluate patients’ participation, satisfaction, and impression of change.

## Methods/design

### Study design

The impact and benefit of the PEP will be evaluated by comparing the educational approach and the “conventional” management of pain. The Step 5 of the EFFADOL project is a multicentre, stepped-wedge, cluster randomised controlled trial. This particular randomised design known as the step-wedge procedure [17–19] minimize the risk of contamination between the two groups (conventional vs TPE approach) and thereby the risk of bias. Indeed, when the purpose is to compare two practices (in this case, TPE and conventional care) in which the attitudes of the caregivers are changed, it is critical to set up at the same time, and with the same health staff the two assessed different modes of care. The stepped-wedge design particularly suits in such setting since it makes it possible to stagger the training of the caregivers hospital by hospital and consequently that of the educational intervention per participating centre. The randomisation is performed at the cluster level, instead of the patient level.

Thus, 6 clusters will be formed in which TPE dispensing will be strictly identical. The first cluster includes 11 participating centres from Basse-Normandie where enrolled patients will all receive the educational approach as healthcare (physician/nurse) staff at the regional level have been already trained in TPE (Step 1 of the EFFADOL project). Then, five other clusters that correspond to five participating centres outside the region at the national level will be gradually included in a stepped-wedge design (Fig. 1). Finally, the conventional approach (before training) will be compared to the educational approach (after being trained).

**Fig. 1:** Schematic representation of the stepped-wedge design

### Study sites

Participating sites include eleven structures from Basse-Normandie (Centre Hospitalier Aunay-Bayeux; Centre Hospitalier Universitaire, Caen; Centre François Baclesse, Caen; Polyclinique du Parc, Caen; Centre Hospitalier, Lisieux; Centre Hospitalier Avranches-Granville; Centre Hospitalier, Cherbourg; Centre Hospitalier, Saint-Lô; Centre Hospitalier Intercommunal, Alençon-Mamers; Centre Hospitalier, Argentan; Centre Hospitalier, Flers) and five structures outside Basse-Normandie (Gustave Roussy, Villejuif; Centre Oscar Lambret, Lille; Centre Hospitalier, Dieppe; Groupement Hospitalier Public Sud de l’Oise, Senlis; Centre Hospitalier Universitaire, Brest).

### Study population

Eligibility criteria are detailed in Table 1. More specifically, pain-related criteria are based on the definition of unbalanced background pain according to the Standards, Options and Recommendations [20]. Briefly, the targeted patients had to experience pain related to disease or its treatments, pain during the previous week, pain intensity greater or equal to 4 on a scale of 10, or pain stopping them from sleeping, or more than 4 episodes of paroxysmal pain per day, or an impact or their daily activities.

**Table 1:** Study eligibility criteria

Inclusion criteria	- Patient suffering from a cancer diagnosed since at least 1 month - Pain related to the pathology or its treatment and/or to the sequelae of disease and its treatment (ongoing or not): - treated with analgesics since at least 1 month - moderate to severe intensity, unbalanced, in the previous week: • Pain intensity ≥4 (on a 0–10 numerical rating scale) • OR leading to insomnia • OR > 4 daily breakthrough pain • OR interference with daily activities - Patient with a life expectancy ≥6 months - Health compatible with the PEP requirements (WHO performance scale ≤2) - Patient with a signed informed consent before inclusion of the study - Patient ≥18 years old - Patient able to understand, speak and read French - Patient without cognitive dysfunctions
Exclusion criteria	- Primary central nervous system cancer or brain metastases - Documented cognitive disorders - Progressive psychiatric disease - Drug user - Heavy drinking, superior to the WHO recommendations - Patient refusal to participate

### Study flowchart

For all the participants with signed consent form, assessments will be conducted at baseline and 8 weeks after inclusion (Fig. 2). For patients of the experimental PEP group, complementary assessments will be performed twice during the program.

**Fig. 2:** Study flowchart. Abbreviations: PEP Pain Education Program

### Assessments

Validated questionnaires and scales used for assessments are presented in Table 2. At inclusion, previous medical history will be reported as well as relevant indications (cancer and pain data, analgesic treatment…).

**Table 2:** Questionnaires and scales used to assess pain, educational impact and satisfaction with the PEP

^1^ Questionnaires will be filled during a visit to hospital or sent by post

^2^ At inclusion

^3^ For control patients, questionnaires will be addressed 8 weeks after inclusion

*Abbreviations: PEP* Pain Education Program

#### Assessment of pain and its impact, and evaluation of analgesic treatment adherence

The “Questionnaire concis sur les douleurs”, corresponding to the validated French translation of the Brief Pain Inventory (BPI, [21, 22]), is very commonly used in research protocols [9]. It allows a rapid self-assessment of the impact of pain on daily activities, using 7 items (general activity, mood, walking ability, normal work, relations with other people, sleep, and enjoyment of life). The use of subscale 9 is therefore recommended by the French National Authority for Health (HAS) to assess QoL in patients suffering from pain [23]. The BPI will be also used to calculate the Pain Management Index (PMI), which, combining intensity and analgesic treatment, can assess the proper use of analgesics [24]. Moreover, adherence to analgesic drugs will be assessed with a pain-adapted questionnaire.

Among the other criteria (assessed only in PEP group), emotional repercussions will be assessed by the Hospital Anxiety and Depression Scale (HADS, [25] and the qualitative assessment of pain will be measured by the short form of the McGill Pain Questionnaire [26] in its French version (Questionnaire de Saint-Antoine (QDSA), [27]).

#### Assessment of the educational dimension of the PEP

Patient’s acquisition of knowledge and skills about his/her pain and treatment will be assessed using a questionnaire developed by our working group and administered at the beginning and at the end of the PEP. Scales evaluating the patient’s self-efficacy to participate actively in pain management and to communicate optimally with caregivers will be also used [28]. The patient’s feeling of changes in his health and its repercussion following the PEP will be retrospectively assessed using sensitive scales [29] particularly adapted to pain.

#### Assessment of participants’ satisfaction and educators’ satisfaction with the PEP

Standards tools recommended by the HAS will be adapted to cancer pain on the basis of those proposed by PLANETH Patient (Plateforme Normande d'Education Thérapeutique du Patient), a regional body whose particular mission is to harmonise TPE practices and their evaluation [30]. The questionnaires deal with the modalities of the workshops (duration, frequency), the benefits of pain management, the quality of the educators and their ability to efficient communication.

The assessment of the program and its benefits for patients will be also conducted with the caregiver-educators. It will evaluate the PEP impact on the educational team in terms of functioning, changes in practices and incorporation with the offer of local care, including communication with the attending physician.

#### Assessments addressed to the patients’ relatives

Patients’ relatives willing to participate to the PEP will have their own QoL evaluated by a self-questionnaire specifically developed in oncology and validated in French (CarGoQoL, [31]). Analgesic treatment adherence, assessment of knowledge and skills about patients’ pain and treatment, and satisfaction with the PEP will be evaluated in relatives using similar questionnaires which have been adapted to them.

#### Primary and secondary endpoints

The main judgement criterion in this study is the impact of pain on daily activities measured with the BPI. A score will be established by averaging the response on the 7 items of the subscale 9. The benefit of TPE on the impact of pain will be defined as a 2-point-decrease (on a scale of 10) between the values measured before and at the end of the PEP (at 8 weeks after inclusion). A 2-point decrease on the BPI scale correspond to a clinically significant improvement [32].

The first secondary endpoint is the proportion of patients adhering to the whole PEP (3 sessions), adherence being defined as the achievement of these 3 sessions for patients who undertook to follow them.

Other secondary endpoints are based on:

- Pain intensity and relief (BPI), its impact on QoL (subscale 9 of BPI, HADS), qualitative characteristics of pain (QDSA) and pain adherence.

- Patient’s knowledge and skills about pain, patient’s self-efficacy to actively manage pain, patient-reported impression of improvement.

- Participants’ satisfaction and educators’ satisfaction with PEP.

### Statistical analysis

#### Sample size calculation

The calculation of the number of subjects needed for statistical significance is based on the main judgement criterion and on the first secondary endpoint.

To meet the first primary objective (Step 5 of the study) building on a stepped-wedge design, the calculation of needed number of patients is based on a ≥ 2-point decrease of the mean score of the BPI subscale 9 at 8 weeks after inclusion, in the experimental PEP group compared to the control group (corresponding to a clinically significant improvement). The calculation takes into account that randomisation is done by clusters (patients belonging to a same cluster are not independent). Based on bilateral test and common-factor variances (2.5-point standard deviation in both groups (intraclass correlation coefficient = 0.05; 3 clusters per randomisation arm; alpha = 5%; power = 80%) it is estimated that 45 patients per arm equitably distributed between the 6 clusters, for a total of 90 assessable patients (Fig. 3).

**Fig. 3:** Expected distribution of patients according to the stepped-wedge design

Moreover, all 5 participating regions outside Basse-Normandie candidates for training their caregivers to TPE, will each include 15 assessable patients in the control group (before being trained). It will be therefore possible to compare, at the region scale, the effect of TPE implementation on daily activities.

To meet to the objective of the Step 4, the judgement criterion is the proportion of patients recruited in Basse-Normandie area adhering to the whole PEP.

Under the assumptions of p_0_ = 0.70, p_1_ = 0.85, α = 5%, and β = 10%, 80 patients are necessary (unilateral exact binomial test that compares a proportion to a reference value) in order to best characterize adhesion to the PEP in the region (Fig. 3).

Of these patients, 15 will be randomly assigned for participation of Basse-Normandie in the primary objective (Step 5 of the study).

Overall, 230 evaluable patients are required; it is therefore planned to recruit 260 patients in order to anticipate some non-assessable patients.

#### Data analysis

At every stage of the analysis, exploratory data will provide, for quantitative variables, mean, its standard deviation, median, quartiles, and missing data; for qualitative variables, frequencies and 95% confidence interval. Statistical tests and confidence intervals will be calculated with an overall error significance level of 5%. For the main objective (Step 5), statistical analysis will be done on the per-protocol population: it will concern assessable patients who have completed the whole program (3 sessions after the educational diagnosis).

Pain interference with daily life scores at 8 weeks post inclusion will be first compared between experimental PEP group and control group, in consideration of the correlation of data (generalized linear mixed model).

For the first secondary objective (Step 4), patients’ adherence to the PEP at the regional scale will be assessed using one-sided test comparing a proportion to a reference value.

For all the steps, a global analysis will be performed, taking into account the different periods of the study, clusters, and the care provided for each period, using a generalized linear mixed model for scales scores and for qualitative results obtained from questionnaires. This analysis will be adjusted to the patients’ demographic and clinical characteristics.

#### Internal validity of the methodology

The choice of the BPI subscale 9 as main endpoint is based on different scientific arguments.

BPI-sf is one of the most widely used pain assessment instrument. Besides pain severity, this questionnaire evaluates the impact on interference. The IMMPACT (Initiative on Methods, Measurement, and Pain Assessment in Clinical Trials) panel recommended that this criterion should be included in all chronic-pain clinical trials [33, 34]. This consensus panel specifically identified the interference items of BPI as one of the scales recommended for the assessment of pain-related functional impairment [35] with a high reliability (*Cronbach alpha reliability ranges from 0.77 to 0.91*). It has been translated and validated in French [22] and the subscale 9 has been recommended by the HAS to assess pain interference with daily life [23].

## Discussion

Nearly one of two patients with cancer pain is undertreated [36]. Patients’ attitudinal barriers in cancer pain remain frequent and are associated with less pain control [37]. Active patient involvement and self-management education appears to be a relevant approach in this regard [38].

In this context, we developed a 5-step project responding to some objectives of the regional health policy and of to third French cancer plan [39]. The construction of a regional PEP, after healthcare staff training to TPE, was based on prior identification of patients’ educative needs regarding cancer pain. PEP implementation will be evaluated through two research steps, first on a regional scale and then on a national one, object of the present study.

In clinical trials, RCT are considered the gold standard of evaluation and as such are mainly used to validate the impact of PEP [10, 38]. The recent systematic review of Oldenmenger et al. [10] reported an improvement in pain intensity in 31% of the PEP studies. The authors incriminate the possible contamination of the control group which could lead to underestimate the actual effect of PEP. In this project, a particular design known as the stepped-wedge procedure was chosen since it allows in particular to provide some control of confounding factors through cluster randomisation [40].

This paper therefore presents the design of a stepped-wedge cluster randomised controlled trial to investigate the effectiveness of TPE in improving cancer pain self-management. The impact and benefit of PEP will be evaluated by comparing the educational approach and the “conventional” management of pain.

The most commonly used criteria to evaluate pain improvement in PEP is pain intensity [9]. Nevertheless, assessment of pain interference with daily life was retained as main endpoint in this study as it appears to less fluctuant and more realistic. Pain interference constitutes in this regard a relevant measure of enhancement in QoL, the latter being the ultimate goal of TPE.

We also took a special interest in educational specifically addressed parameters. Besides patients’ knowledge and attitudes, patients’ communication skills and active participation in their pain management will be assessed.

Satisfaction with treatment might act as a contributor to other outcomes and encourages patient involvement in pain management. Patient satisfaction with cancer pain care strongly correlates with retrospective ratings of overall improvement [29]. Patient-reported improvement scale will be retrospectively measured following the PEP in order to assess the patient’s feeling of changes in his health as well as a clinically significant change.

In addition, evaluation of participants’ and educators’ satisfaction with the program will be used to further optimize the latter by adjusting the followed procedures in necessary.

In conclusion, the originality and strength of this project are based on collaborative work between healthcare professionals and a research approach building on robust methodologies that seek to demonstrate the effectiveness of TPE in improving the patients’ skill in cancer pain management. Dissemination of this educational approach (at regional and then national level) will likely be accompanied by a long term change in practices that should provide mutual benefit to patients and caregiver-educators.

Besides the benefit of PEP for individuals, cancer pain is a national challenge and better managing it is a major public health issue. In this regard, TPE, by giving an impetus to changing patterns of behaviors and attitudes, constitutes an asset to allow better assessment, treatment, and understanding of the problem.

## Data Availability

Not applicable.

## Abbreviations

BPI: Brief Pain Inventory
EFFADOL: *Ensemble, Faire FAce à la Douleur*
ERET: *Espace Régional d’Education Thérapeutique*
HADS: Hospital Anxiety and Depression Scale
HAS: French National Authority for Health
PEP: Pain Education Programs
QDSA: Questionnaire de Saint-Antoine
QoL: Quality of Life
RCT: Randomised Controlled Trials
TPE: Therapeutic Patient Education
WHO: World Health Organization

## References

[1] Portenoy RK, Ahmed E (2014). Principles of opioid use in cancer pain. J Clin Oncol.

[2] Van den Beuken-van Everdingen MHJ, Hochstenbach LMJ, Joosten EAJ, Tjan-Heijnen VCG, Janssen DJA (2016). Update on prevalence of pain in patients with Cancer: systematic review and meta-analysis. J Pain Symptom Manag.

[3] Kroenke K, Theobald D, Wu J, Loza JK, Carpenter JS, Tu W (2010). The association of depression and pain with health-related quality of life, disability, and health care use in cancer patients. J Pain Symptom Manag.

[4] Greco MT, Roberto A, Corli O, Deandrea S, Bandieri E, Cavuto S (2014). Quality of cancer pain management: an update of a systematic review of undertreatment of patients with cancer. J Clin Oncol.

[5] Ward SE, Goldberg N, Miller-McCauley V, Mueller C, Nolan A, Pawlik-Plank D (1993). Patient-related barriers to management of cancer pain. Pain..

[6] Brant JM (2010). The global experience of cancer pain. Asian Pac J Cancer Prev.

[7] Kwon JH (2014). Overcoming barriers in cancer pain management. J Clin Oncol.

[8] World Health Organization. Regional Office for Europe (1998) Therapeutic patient education: continuing education programmes for health care providers in the field of prevention of chronic diseases: report of a WHO working group. Copenhagen: WHO Regional Office for Europe. [http://www.euro.who.int/__data/assets/pdf_file/0007/145294/E63674.pdf]. Accessed 20 June 2019.

[9] Prevost V, Delorme C, Grach MC, Chvetzoff G, Hureau M (2016). Therapeutic education in improving Cancer pain management: a synthesis of available studies. Am J Hosp Palliat Care.

[10] Oldenmenger WH, Gearing JI, Mostovaya I, Vissers KCP, de Graeff A, Reyners AKL (2018). A systematic review of the effectiveness of patient-based educational interventions to improve cancer-related pain. Cancer Treat Rev.

[11] Adam R, Bond C, Murchie P (2015). Educational interventions for cancer pain. A systematic review of systematic reviews with nested narrative review of randomized controlled trials. Patient Educ Couns.

[12] Bennett MI, Bagnall AM, José Closs S (2009). How effective are patient-based educational interventions in the management of cancer pain?. Pain..

[13] Cummings GG, Olivo SA, Biondo PD, Stiles CR, Yurtseven O, Fainsinger RL (2011). Effectiveness of knowledge translation interventions to improve cancer pain management. J Pain Symptom Manag.

[14] Jho HJ, Myung SK, Chang YJ, Kim DH, Ko DH (2013). Efficacy of pain education in cancer patients: a meta-analysis of randomized controlled trials. Support Care Cancer.

[15] Prevost V, Clarisse B, Heutte N, Leconte A, Bisson C, Bignon R (2018). Therapeutic patient education in Cancer pain management: from practice to research: proposals and strategy of the French EFFADOL program. J Cancer Educ.

[16] Prevost V, Delorme C, Heutte N, Leconte A, Bechet C, Licaj I, Bignon R, Bisson C, Cauchin S, Gicquère M, Grach MC, Guillaumé C, Le Garrec J, Ropartz MC, Roux N, Sep Hieng V, Le Chevalier A, Clarisse B. Evaluation of patients’ needs to design and assess a patient education program in cancer pain. J Pain Res. 2019;12:1813–23.10.2147/JPR.S197920PMC656018431239759

[17] Rasmussen CD, Holtermann A, Mortensen OS, Søgaard K, Jørgensen MB (2013). Prevention of low back pain and its consequences among nurses' aides in elderly care: a stepped-wedge multi-faceted cluster-randomized controlled trial. BMC Public Health.

[18] Hussey MA, Hughes JP (2007). Cluster randomized crossover trials: design and analysis of the stepped wedge design. Contemp Clin Trials.

[19] Mdege ND, Man MS, Taylor CA, Torgerson DJ (2011). Systematic review of stepped wedge cluster randomized trials shows that design is particularly used to evaluate interventions during routine implementation. J Clin Epidemiol.

[20] Poulain P, Michenot N, Ammar D, Delorme C, Delorme T, Diquet B (2012). Mise au point sur l’utilisation du fentanyl transmuqueux chez le patient présentant des douleurs d’origine cancéreuse (version longue). Doul et Analg.

[21] Cleeland CS, Ryan KM (1994). Pain assessment: global use of the brief pain inventory. Ann Acad Med Singap.

[22] Larue F, Colleau SM, Brasseur L, Cleeland CS (1995). Multicentre study of cancer pain and its treatment in France. BMJ..

[23] ANAES, Evaluation et suivi de la douleur chronique chez l’adulte en médecine ambulatoire, Service des Recommandations et Références professionnelles, février 1999. [http://www.has-sante.fr/portail/upload/docs/application/pdf/douleur1.pdf]. Accessed 20 June 2019.

[24] Zelman D. C., Cleeland C. S., Howland E. W. (1987). Factors in appropriate pharmacological management of cancer pain: A cross-institutional investigation. Pain.

[25] Razavi D, Delvaux N, Farvacques C, Robaye E (1990). Screening for adjustment disorders and major depressive disorders in cancer in-patients. Br J Psychiatry.

[26] Boureau F, Luu M, Doubrère JF (1992). Comparative study of the validity of four French McGill pain questionnaire (MPQ) versions. Pain..

[27] Marquié L, Duarte L-R, Mauriès V, Izard P, Pouymayou J (2008). Les caractéristiques psychométriques du Questionnaire de douleur de Saint-Antoine en consultation d’algologie chez les personnes atteintes de cancer. Doul et Analg..

[28] Street RL, Slee C, Kalauokalani DK, Dean DE, Tancredi DJ, Kravitz RL (2010). Improving physician-patient communication about cancer pain with a tailored education-coaching intervention. Patient Educ Couns.

[29] Fischer D, Stewart AL, Bloch DA, Lorig K, Laurent D, Holman H (1999). Capturing the patient’s view of change as a clinical outcome measure. JAMA..

[30] PLANETH Patient (Plateforme Normande d'Education Thérapeutique du Patient). Evaluation quadriennale. [http://www.planethpatient.org/evaluation-quadriennale]. Accessed 20 June 2019.

[31] Minaya P, Baumstarck K, Berbis J, Goncalves A, Barlesi F, Michel G (2012). The CareGiver oncology quality of life questionnaire (CarGOQoL): development and validation of an instrument to measure the quality of life of the caregivers of patients with cancer. Eur J Cancer.

[32] Cleeland CS, Body JJ, Stopeck A, von Moos R, Fallowfield L, Mathias SD (2013). Pain outcomes in patients with advanced breast cancer and bone metastases: results from a randomized, double-blind study of denosumab and zoledronic acid. Cancer..

[33] IMMPACT (Initiative on Methods, Measurement, and Pain Assessment in Clinical Trials). [http://www.immpact.org/]. Accessed 20 June 2019.

[34] Dworkin RH, Turk DC, Farrar JT, Haythornthwaite JA, Jensen MP, Katz NP (2005). Core outcome measures for chronic pain clinical trials: IMMPACT recommendations. Pain..

[35] Dworkin RH, Turk DC, Wyrwich KW, Beaton D, Cleeland CS, Farrar JT (2008). Interpreting the clinical importance of treatment outcomes in chronic pain clinical trials: IMMPACT recommendations. J Pain.

[36] Deandrea S, Montanari M, Moja L, Apolone G (2008). Prevalence of undertreatment in cancer pain. A review of published literature. Ann Oncol.

[37] Gunnarsdottir S, Sigurdardottir V, Kloke M, Radbruch L, Sabatowski R, Kaasa S (2017). A multicenter study of attitudinal barriers to cancer pain management. Support Care Cancer.

[38] Howell D, Harth T, Brown J, Bennett C, Boyko S (2017). Self-management education interventions for patients with cancer: a systematic review. Support Care Cancer.

[39] Institut National du Cancer- Plan cancer 2014-2019 : priorités et objectifs [http://www.e-cancer.fr/Plan-cancer/Plan-cancer-2014-2019-priorites-et-objectifs]. Accessed 20 June 2019.

[40] Hemming K, Haines TP, Chilton PJ, Girling AJ, Lilford RJ (2015). The stepped wedge cluster randomised trial: rationale, design, analysis, and reporting. BMJ..

